The article "Synthesis of Molecularly Imprinted Cryogels to Deplete Abundant Proteins from Bovine Serum" was published in 2018. Journal: Polymers (Basel).

# Synthesis of Molecularly Imprinted Cryogels to Deplete Abundant Proteins from Bovine Serum

**DOI:** 10.3390/polym10010097

**Published:** 2018-01-20

**Authors:** Chun Yang, Yan Zhang, Wei-Qin Cao, Xiao-Feng Ji, Jian Wang, Ya-Nan Yan, Tao-Lin Zhong, Yu Wang

**Affiliations:** School of Chemistry & Chemical Engineering, Yangzhou University, 180 Siwangting RD, Yangzhou 225002, China; m18852727909@163.com (Y.Z.); Amber612_qin@163.com (W.-Q.C.); MX120170303@yzu.edu.cn (X.-F.J.); wjian@yzu.edu.cn (J.W.); M150323@yzu.edu.cn (Y.-N.Y.); 18852721427m@sina.cn (T.-L.Z.); ycwangyu@yeah.net (Y.W.)

**Keywords:** molecularly imprinted polymer, cryogel, bovine serum, abundant protein, depletion

## Abstract

Molecularly imprinted polyacrylamide cryogels were synthesized with pending templates (bovine serums of different concentrations). As the serum concentrations increased in the monomer solutions, the resulting cryogels could adsorb and deplete more proteins from serum samples. Due to the addition of vinyltriethoxysilane (VTEOS) in the prepolymerizing solutions, the polymers came as organic–inorganic hybrid materials. It endued the silica-modified amphoteric polyacrylamide cryogels with improved mechanical strengths. Scanning electron micrography (SEM), Infrared (IR) spectrometry, thermogravimetry-differential thermal analysis (TG-DTA), and X-ray photoelectron spectroscopy (XPS) were carried out to characterize these macroporous polymers. Amphoteric cryogels proved to be favorable materials recognizing and binding proteins. When used as liquid chromatography stationary phases, they were capable of simultaneously adsorbing various serum proteins. Electrophoresis showed that abundant proteins were gradually depleted by the cryogels prepared from increased ratios of bovine serums in the monomer solutions. As abundant proteins are always imprinted first, this sample per se imprinting method provides an effective and convenient way to deplete abundant proteins from complex samples such as serums, meanwhile concentrating and collecting scarce species therein.

## 1. Introduction

Molecularly imprinted polymers (MIPs) are synthesized to achieve specific interactions and mutual responses between the polymeric matrices and the related templates [1,2]. Those stable polymeric materials possess amazing properties and functions by bearing predetermined exclusive binding sites against certain target molecules (templates). After extensive research and development of more than 40 years, MIPs have not only attracted considerable research interests in scientific communities [3], but also set out on a journey to industrial purposes [4]. At present one can easily find the application of MIPs in various fields [5,6,7] for different applications such as separation [8], purification [9], catalyzing [10], sensoring [11], etc.

Proteins are of great academic and industrial importance. There has been unprecedented enthusiasm for the topic of molecular recognition and interaction involving proteins. Through rationally designed synthetic methods, people expected to get robust polymers mimicking antibody [12] or enzyme-like selectivity and affinity [13]. Unfortunately the field of protein imprinting has seen limited success to generate that type of artificial biomimetic materials [14]. To overcome the inherent huge resistance of mass transfer related to macromolecules, protein imprinting usually counts on low-dimensional techniques, i.e., imprinting on surfaces or nanoparticles [15].

Cryogenic polymerization proceeds at sub-zero temperatures. When water was used solely or a suitable portion of the solvents, a procedure of freezing-swelling-thawing produces macroporous polymers known as cryogels [16]. Macropores of more than 100 μm in these polymers can facilitate internal mass transferring, greatly favoring the treatment of biomacromolecules [17]. In order to fully explore this advantage, more and more protein-imprinted cryogels have been synthesized and studied. Ice crystal squeezing effects not only influence skeleton structures but also manipulate the stacking layout of chemical groups in cryogels. Besides conventional functions such as protein recognition [18,19,20,21], purification/separation [9,22,23,24], or depletion [25], cryogels could be prepared to act as catalysts [26] and fluorescent materials [27].

Being encountered with diverse target molecules, an alternative proteomic methodology should hold an extensive adaptability to complicated samples from various organisms. Here we report the synthesis of molecularly imprinted cryogels with different ratios of bovine serums as pending templates. Liquid chromatography columns made of these cryogels possess specific affinities against abundant proteins in the bovine serum, bringing out longer retention time for them than for non-imprinted proteins. Finally, the depletion of the abundant proteins was testified by a polyacrylamide gel electrophoresis experiment of the eluates from those cryogel columns. From now on one can deplete abundant proteins based on the intrinsic properties of a complex sample rather than any extrinsic assistance. To some degree, sample understanding seems unnecessary, because it is an efficient and low-cost method achieved by feeling free to perform molecular imprinting against sample heterogeneities.

## 2. Experimental Section

### 2.1. Instruments and Reagents

Acrylic acid, diallylamine, acrylamide (AM), *N*,*N*-methylenebisacrylamide (BisAM), and vinyltriethoxysilane were purchased from Haopeng Chemical Plant (Jinan, Shandong, China). Coomassie brilliant blue R250, *N*,*N*,*N*,*N*-tetramethyl ethylenediamine (TEMED), boric acid, sodium hydrogen sulfite (SHS), sodium dodecyl sulfate (SDS), and ammonium peroxydisulfate (APS) were purchased from Sinopharm Chemical Reagents Co., Ltd. (Shanghai, China). Bovine serum (fetal calf serum) was purchased from Zhejiang Tianhang Biotechnology Co., Ltd. (Deqing, Zhejiang, China). All other chemicals were of analytical reagent grade.

Morphology of the polymers was characterized by SEM (S-4800, Hitachi, Tokyo, Japan). The thermal stability of polymers was tested with thermal gravimetric-differential thermal analysis (Pyris 1 TGA, PerkinElmer Co., Ltd., Shelton, CT, USA) at a rate of 10.0 °C/min from 30.0 °C to 800.0 °C under a nitrogen flow of 20.0 mL/min. Binding energies were measured with an X-ray photoelectron spectrometer from ThermoFisher Scientific (ESCALAB 250Xi, Waltham, MA, USA). Infrared characterization was carried out on a microscopic IR spectrometer (670-IR, Varian, Palo Alto, CA, USA).

### 2.2. Preparation of Modified Polyacrylamide Cryogels

Bovine serum proteins imprinted cryogel were synthesized according to previously reported methods [28,29]. The synthesis of 1 non-imprinted polymer (NIP) and 4 MIPs followed an identical protocol and carried out simultaneously to exclude external influences on the performance of the polymers (Table 1). Each cryogel was made from a solution containing an equivalent of monomers and initiator but different amount of bovine serum. In brief, SHS, acrylamide (AM), *N*,*N*-methylenebisacrylamide (BisAM), acrylic acid, and vinyltriethoxysilane were stirred and dissolved in water. After the addition of bovine serum, diallylamine was then introduced. Both before and after the addition of APS, the solutions were ultrasonically degassed for 3 min respectively. Finally, the resultant mixtures were transferred into plastic bags. Cryogenic polymerization was carried out by putting the monomer solutions in a refrigerator at −20 °C for 24 h. Besides imprinted cryogels, an NIP was synthesized at the same time for comparison (Table 1).

All cryogels were thawed in a water bath at 50 °C for 2 h before washing. Unreacted monomers and inorganic salts were directly washed with deionized water. To remove template molecules, the MIPs were put in a ultrasonic cleaner and washed with 1 M NaCl (containing 5 g/L SDS) for five times (20 min each), till the absorbance of the scrubbing solution was minimized at 278 nm. All the MIPs and the NIP were dried at 60 °C for 6–8 h before further use.

### 2.3. Conductometric Titrations of the Amphoteric Cryogels

As the amounts and densities of the amino and carboxyl groups greatly affect protein imprinting. It is necessary to quantify the functional groups on the cryogels. The amount of arboxyl or amino was determined by a conductometric titration method [29] with a DDS-11 digital conductometer (Falanduo Technology Development Co., Ltd., Shanghai, China).

### 2.4. Protein Adsorption on the Cryogels

Adsorption kinetics and adsorption capacities of serum proteins on the polymers were measured with a UV–Visible spectrophotometer at 278 nm (UA2550, Shimadzu, Kyoto, Japan). To investigate the adsorption kinetics, 0.05 g of cryogels were added in a centrifuge tube with 10 mL solution of bovine serum (diluted with 20 times volume of water). The protein concentrations were measured after shaking the centrifuge tubes at room temperature for different time intervals. Adsorption capacities (*Q*, mg/g) of bovine serum proteins were determined similarly after saturation (shaken at room temperature for 6 h), and calculated according to the following equation:

*Q* = (*C*_0_ − *C_t_*)*V/m* (1)

where *C*_0_ and *C_t_* represent the initial and equilibrium protein concentrations respectively. *V* is the volume (mL) of the solution, and *m* is the dry weight of the polymer (g). *C*_0_ was determined based on a calibration curve of Coomassie brilliant blue G250 dyed BSA at 595 nm.

### 2.5. High Performance Liquid Chromatography (HPLC)

Dried cryogels were ground into small homogeneous particles of less than 0.5 mm and loaded in 2 cm stainless tubes as liquid chromatography (LC) stationary phases. HPLC was performed on a 1200 HPLC Series system of Agilent Technologies (Santa Clara, CA, USA). A phosphate buffer (0.1 M, pH = 7.20) was used as the mobile phase at a flow rate of 0.1 mL/min. Each time a serum solution of 20 μL was injected and detected at a wavelength of 278 nm. The eluates were collected from 0 to 15 min for electrophoresis experiments to check depletion functions.

### 2.6. SDS Polyacrylamide Gel Electrophoresis (SDS-PAGE)

SDS-PAGE was performed on a DYCZ-24DN Electrophoresis System (Liuyi Biological Technology Co., Ltd., Beijing, China) in accordance with a previously reported method [30].

## 3. Results and Discussion

### 3.1. Morphological, Structural and Physicochemical Characterization of Cryogels

Both imprinted and non-imprinted crygeols are polymers very alike in appearance, with macropores around 100 μm (Figure 1). In many aspects the NIP is similar to the molecularly imprinted polymer (MIP) but without specific binding sites for the templates. However, this functional difference is hardly to be seen from either STM or FTIR. Occasionally the serum-imprinted cryogels were slightly dyed yellowish, nonetheless that did not invalidate their functions to recognize and bind proteins. After the removal of its protein templates, an imprinted cryogel provides an IR spectrum (Figure 2a) very similar to that of the NIP (Figure 2b). It clearly shows that either the MIP or the NIP shares quite analogous molecular structures, vibrations and rotations from same functional monomers.

Generally cryogel materials are stable under ambient and conventional service conditions. From room temperature to 227.5 °C under the protection of a nitrogen flow, a cryogel just lost 6.9% of its mass (Figure 3), which very likely presents the volatilization of absorbed water. Material decomposition began above 228 °C and the polymer started to release small molecules such as water and ammonia. Afterwards obvious carbonization happened at 338 °C, the cryogel lost most mass before 800 °C.

Vinyltriethoxysilane was added in the monomer solutions to prepare organic-inorganic hybrid polymers. The existence of silicon could be observed in Figure 4. It is expected that the hydrolysis of the siloxane led to interpenetrated silica textures in the polymers. Organic-inorganic structures will properly improve the mechanical strengths for the cryogels, making them better stationary phases for HPLC experiments.

In the conductometric titration, NaOH was used to neutralize carboxyl groups. As the titrant added in, the ionization of the acidic groups enhanced the electrical conductivity of the solution containing the polymer. It produces gradually ascending titration curves for both the MIP and the NIP (Figure 5). However polymerization did not progress synchronously in different solutions. Even from a solution of same composition, the MIP (Figure 5a) consumes less titrants than the NIP (Figure 5b). Accordingly the acidic group densities were calculated 1.3 mmol/g (RSD 7%) for the MIP, and 1.6 mmol/g (RSD 6%) for the NIP.

Unexpectedly amino densities on the cryogels could not be determined in the same way. Possibly due to an inferior reactivity of diallylamine, there were not adequate amino groups solidified in the polymers. All the titration curves of protonized amino were flat, not showing clear turning points to confirm stoichiometric points (not included here).

### 3.2. Influencing Factors on Adsorption and Imprinting

It is believed that three-dimensional recognizing cavities have been formed in amphoteric cryogels against protein templates. To accomplish specific recognitions for macromolecules or bigger things such as cells, one should fully consider templates about the imprinting-influenced factors such as shape, size and charges. They must be made not only to approximately fill the cavity shapes [31,32], but also to correspond to the interfacial charged groups with their own surface ionized groups [33,34]. Certainly it is preferable to take both shape and charge into account at the same time [29,33]. However, multiplex-site recognitions of various mechanisms would inevitably lead to slow kinetics including both molecular migration and orientation. As a result, protein adsorption on the NIP is faster than that on the MIP (Figure 6a). In a solution of bovine serum diluted with a same volume of water, it reaches an adsorption equilibrium for the NIP in 2.5 h. In regard to the MIP, protein adsorption was saturated 3 h later (Figure 6b).

As main monomers utilized in the polymerization reactions, AM and BisAM are dominating elements to build the cryogel skeletons. With the foundational structures of cross-linked polyacrylamide, cryogels are efficacious to manipulate proteins through weak forces such as hydrogen bonds, hydrophilic and hydrophobic interactions. In order to enhance the mutual adaption of the polymers and templates, both acrylic acid and diallylamine were introduced. An order of magnitude stronger coulombian forces therefore worked between the ionized functional groups of the polymers and proteins. It is necessary to point out that the added volumes of the unsaturated acid and amine are very crucial to adjust the recognizing powers of the polymers. A small quantity of acrylic acid and diallylamine did enhance the recognition specificity to a protein by orientationally anchoring its surface ionized amino acid residues [29]. Overmuch or inadequate addition of charged monomers could weaken recognizing powers, but better than non-amphoteric cryogels made from just AM and BisAM. In addition, it is found that protonated allylamine indicated a higher polymerization activity. Hence acrylic acid was added more to efficiently polymerize the amine (Table 1).

Here prepared cryogels, either the NIP or MIPs, have higher adsorption capacities than that previously reported [30]. Based on imprinting-induced specific binding sites, the MIP adsorbs much more protein templates than the NIP (Figure 7). Calculation according to equation 1 reveals that the adsorption capacities are 160.4 mg/g for the MIP and 14.2 mg/g for the NIP. Accordingly, the imprinting factor (IF) was calculated as the value of *Q_MIP_*/*Q_NIP_* = 11.3, which is also higher than that of the MIPs previously reported. As a whole, the imprinted cryogels do not adsorb much protein, in the region of several hundreds mg per gram polymer. However the adsorption of the MIP is overwhelmingly based on specific recognition. This makes imprinted cryogels preferable materials in proteomic applications.

### 3.3. Chromatography and Electrophoresis Results

Hybrid materials usually benefit from both the organic and inorganic moieties. That is why we introduce a siloxane monomer in the prepolymerizing solutions to synthesize the protein-imprinted cryogels.

Vinyltriethoxysilane works in two ways during the preparation of the cryogels. Firstly, it acted as a monomer in the polymerization and made the functional group of siloxane be tethered to polymer chains. Secondly the hydrolysis of the siloxane formed local silica structures within the cryogels. As a half more VTEOS was added in the monomer solutions (Table 1), it is expected to achieve improved mechanical strengths for the resulting polymers. In fact, the columns made from these cryogels were more durable than the those previously reported [30].

On the column made of the NIP, all proteins show very short retention time less than 2 min (Figure 8a). It means the retention of the proteins is based on nonspecific adsorption of the low mass transfer resistance polymer. In the case of an MIP column, there are selective recognizing cavities for the imprinted proteins (i.e., abundant species). A peak of much longer time (26.2 min) is observed for the abundant proteins (Figure 8b). At the same time, an inconspicuous peak still appears at 2 min on behalf of low-abundance proteins in the bovine serum sample. An obvious difference of the retention time between the imprinted and non-imprinted proteins ensures their complete separation via a chromatographic operation. Consequently, the abundant and scarce proteins can be differentiated and collected independently. However, an MIP column made from bovine serum imprinting acts as an NIP column, giving a very fast eluting peak for a human serum sample (insertion in Figure 8).

As shown in Figure 9, the electrophoresis bands of the NIP-dealt serum solution (Lane A) is very similar to that of the untreated bovine serum (Lane B). After the retention on those MIP columns, the components of the eluates are quite different. Generally, there are more and more proteins depleted as the serum volumes increased in the monomer solutions (Lanes C–F in Figure 9). If bovine serum was added just as 1/20 to 1/10 volume of the monomer solutions, the MIPs did not exhibit obvious depletion effects. Lanes C and D just show mild depletion of the molecular weight range around 80 k (Figure 9). When 4 mL or more serum were added to get 20 mL solutions (Table 1), the resulting MIPs present notable abilities to remove abundant proteins. Lane F shows a remarkable depletion ability of the 2-fold diluted serum imprinted cryogel. It indicates that the bands of the proteins generating signals around the molecular weight of 170 k, 80 k, 55 k, and 13 k completely disappear. Meanwhile the two bands between 25 and 30 k are more obvious in Lane F than elsewhere. This is believed to be an evidence of enriched rare protein(s) after the depletion of the abundant species.

## 4. Conclusions

Although an optionally allocated mixture of AM, BisAM, acrylic acid and diallylamine is not possibly an optimal choice to imprint any certain template, it is effective for the imprinting of various proteins. When a complex protein sample such as bovine serum was introduced in such a monomer solution, specific recognizing and binding sites were established for proteins in the resulting polymer. The more serum was added, the more specific sites were formed. As the template volume exceeded a threshold proportion, there would be enough adsorptive sites for one or more proteins. With a stationary phase made of such a cryogel, the abundant proteins were completely depleted via a chromatography operation. Additionally, due to their stability, biocompatibility, flexibility and low-cost availability, molecularly imprinted polyacrylamide cryogels are superior materials to manipulate proteins. These MIPs have the potential to play important roles in the fields of proteomic profiling, differential proteomics, biomarker discovery, and so forth.

## Figures and Tables

**Figure 1:** SEM images of (**a**) MIP; and (**b**) NIP.

**Figure 2:** FTIR spectra of (a) MIP and (b) NIP.

**Figure 3:** (**a**) TG and (**b**) DTG curves of cryogel F.

**Figure 4:** XPS of the cyogel F.

**Figure 5:** Conductometric titration curves of (**a**) MIP; and (**b**) NIP.

**Figure 6:** Adsorption dynamic of (**a**) NIP; and (**b**) MIP in bovine serum diluted with 20 times volume of water.

**Figure 7:** Adsorption of serum proteins on (**a**) MIP; and (**b**) NIP at 278 nm. Curve (**c**) is of bovine serum (diluted with 20 times volume of water).

**Figure 8:** Chromatograms of serum proteins on (**a**) NIP; and (**b**) MIP (F in Table 1). Columns: 4.6 mm × 20 mm. Sample: 1/4 diluted bovine serum. Injection volume: 20 μL. Mobile phase: 100 mmol/L PBS (pH 7.20) at 0.1 mL/min. Detection wavelength 278 nm.

**Figure 9:** SDS-PAGE of serum eluates from different columns. (**A**) Diluted original serum; (**B**) NIP, (**C**–**F**) MIP C–F (in Table 1).

**Table 1:** Composition of the monomer solutions.

Reagents	B	C	D	E	F
Bovine serum/mL	0	1	2	4	10
H_2_O/mL	20	19	18	16	10
AM/g	0.5				
BisAM/g	0.3				
Acrylic acid/μL	125				
Diallylamine/μL	63				
VTEOS/μL	150				
SHS/g	0.03				
APS/g	0.06				

AM: acrylamide; BisAM: *N*,*N*-methylenebisacrylamide; VTEOS: vinyltriethoxysilane; SHS: sodium hydrogen sulfite; APS: ammonium peroxydisulfate.
